RETRACTED

# miR-509-5p Inhibits the Proliferation and Invasion of Osteosarcoma by Targeting TRIB2

**DOI:** 10.1155/2019/2523032

**Published:** 2019-12-16

**Authors:** Jiekun Guo, Qiang Wu, Xiaoming Peng, Bin Yu

**Affiliations:** ^1^Department of Orthopedic Surgery, Nanfang Hospital, Southern Medical University, Guangzhou 510515, China; ^2^Department of Orthopedic Surgery, Yuebei People's Hospital, Shantou University, Shaoguan 512026, China

## Abstract

Osteosarcoma (OS) is one of the most common malignant bone tumors in adolescents with a poor prognosis. Though miR-509-5p has been reported as a tumor suppressor in several human cancers, the role of miR-509-5p in OS remains unclear. In this study, our result of real-time PCR (RT-PCR) showed that the expression of miR-509-5p was significantly decreased in OS tissues and cell lines. Overexpression of miR-509-5p significantly suppressed cell proliferation and invasion in OS cell lines. Moreover, we identified tribbles homolog 2 (TRIB2) as the direct target of miR-509-5p. Knockdown of TRIB2 could inhibit the malignant capacity of OS cells. At last, we reported that TRIB2 could inhibit the bioactivity of the tumor suppressor gene p21 via blocking its transcriptional activity. Collectively, our study revealed that miR-509-5p functions as a tumor suppressor by targeting TRIB2 in OS and thus could affect the activity of p21, suggesting that miR-509-5p is a novel preventive intervention for OS patients.

## 1. Introduction

Osteosarcoma (OS) is a highly malignant tumor occurring in children, counting for 3–5% of newly diagnosed cancers of adolescents [1]. Although the five-year survival rate has been improved to 60–75% thanks to the rapid development of treatment strategies, the prognosis remained poor for the complicated carcinogenesis of OS is still unclear [2]. Therefore, it is of great urgency to seek for new biomarkers that targeted preventive and/or therapeutic interventions for OS patients to improve the clinical outcome [3, 4].

MicroRNA (miRNA) is a kind of noncoding RNA with a length of 22–24 nucleotides. It is well recognized that miRNA serves a critical role in the pathological process of various human cancers via binding to the 3′-UTR region of the target gene. Overexpression or low expression of oncogenic or tumor suppressor miRNA is crucial in the progression of tumor development because the miRNA implicates in proliferation, apoptosis [5], autophagy [6], migration [7], and invasion [8]. To date, several miRNAs are reported to play a critical role in the tumorigenesis of OS; for example, miR-182-3p [9], miR-491-3p [10], and miR-376a [11] act as tumor suppressors while miR-33a [12] functions as an oncogene. However, further studies about the relationship between miRNA and OS are still needed for the controversy about the role of the miRNA. Fortunately, the rapid development of the bioinformatic technology brings great convenience for researchers to investigate for a further step.

RETRACTED

In the present study, we explore the impact of miR-509-5p on OS by a series of cellular and molecular function experiments. Then, we performed bioinformatic analysis to predict that TRIB2 was the target gene of miR-509-5p and clarified their relationship by dual luciferase report assay, subsequently. In summary, miR-509-5p functions as a tumor suppressor gene in OS through miR-509-5p/TRIB2 axis, making miR-509-5p a potential diagnostic and/or therapeutic target for OS.

## 2. Materials and Methods

### 2.1. Data Processing

Several GEO databases were used to evaluate the expression of mir-509-5p in osteosarcoma tissues and cell lines. As a result, the expression level of mir-509-5p in osteosarcoma was significantly reduced in GSE28423 relative to paraneoplastic tissue.

Similarly, we found two datasets, GSE39055 and GSE11416, from the GEO website using the “osteosarcoma mRNA” as a search condition and compared the differential genes of different groups using the GEO2R tool that comes with the website. In the GSE39055 dataset, we divided the patients who relapsed within 3 years and the patients who relapsed after 3 years into two groups and obtained a gene set containing 320 differential genes. At the same time, in the GSE11416 dataset, we compared the genes of normal osteoblasts and osteosarcoma cells and obtained a gene set of another 53 differential genes. By taking the above two gene sets, we finally got the target gene TRIB2.

### 2.2. Tissue Collection, RNA Extraction, and Real-Time PCR

15 OS tumor tissues accompanied with their homologous adjacent normal tissues were collected from the patients following surgical resection from January 2017 to March 2019 at the Yuebei People's Hospital, China. No patients received radiotherapy or chemotherapy before surgical resection. All samples were rapidly frozen in liquid nitrogen immediately and stored at −80°C refrigerator until total RNA was extracted. This study was approved by the Yuebei People's Hospital ethical committee and all participants had signed the informed consent.

The total RNA was extracted with Trizol Reagent (Invitrogen, Carlsbad, USA). PrimeScript RT Master Mix (Takara) was used to reverse transcribe 1.0 *μ*g total RNA into a final volume of 20 *μ*l cDNA. The RT-PCR was conducted with the SYBR Select Master Mix (KeyGEN, China), and the subsequent reaction was performed in a QuantStudio 6 Flex Real-Time PCR System as follows: initial denaturation step at 95°C for 10 minutes, followed by 40 cycles at 92°C for 15 seconds and 60°C for 1 minute. The primers used were as follows: GAPDH forward primer, 5′-ATTCCATGGCACCGTCAAGGCTGA-3′; GAPDH reverse primer, 5′-TTCTCCATGGTGGTGAAGACGCCA-3′; miR-509-5p forward primer, 5′-TACTGCAGACAGTGGCAAUCA-3′; miR-509-5p reverse primer, 5′-GTGCAGGGTCCGAGGT-3′; U6 forward primer, 5′-CTCGCTTCGGCAGCACA-3′, U6 reverse primer, 5′-AACGCTTCACGAATTTGCGT-3′.

RETRACTED

### 2.3. Cell Line, Cell Culture, and siRNA Transfection

Four human OS cell lines including U2OS, HOS, Saos-2, MG-63, and normal osteoblast cell line NHOst were purchased from American Type Culture Collection (Manassas, VA, USA). All the cell lines were cultured in Dulbecco's modified Eagle's medium (DMEM; Thermo Fisher Scientific, USA), supplemented with 10% fetal bovine serum (FBS; Thermo Fisher Scientific, USA) and streptomycin (100 *μ*g/ml), penicillin (100 U/ml). The cells were incubated in a 37°C humid incubator containing 5% CO_2_. The culture medium was replaced every 2 days to remove the floating cells and keep the adhering cells for further use.

The U2OS and HOS cells were seeded in six-well plates before transfection. When 60–70% confluence is reached, the cells were transiently transfected with siRNA targeting a specific gene or negative control using Lipofectamine 2000 reagent (Invitrogen, USA). The sequences of the siRNA used above were listed as follows: siRNA-TRIB2: sense 5′-UAGCGAGAUAUGGGAGAUCTT-3′, anti-sense 5′-GAUCUCCCAUAUCUCGCUATT-3′. Si-NC: sense 5′-UUCUCCGAACGUGUCACGUTT-3′, antisense 5′-ACGUGACACGUUCGGAGAATT-3′.

### 2.4. Cell Proliferation Assay

The cell proliferation was investigated by cell counting kit (CCK-8, Biyuntian, Nanjing) assay. Briefly, 3 × 10^3^ cells were planted into a 96-well plate and cultured for 0, 24, 48, 72, and 96 h before 10 *μ*l of CCK-8 reagent was added to the wells. After 2 hours of further incubation protecting from light at 37°C, the absorbance was measured by the microplate reader at 450 nm. All the experiments were repeated 3 times.

### 2.5. Transwell Assay

The invasive ability of the cells was evaluated by the Cell Invasion Assay kit (BD Biosciences, Franklin Lakes, NJ, USA) following the accompanied protocol. A total of 3 × 10^4^ cells were seeded in the upper chamber, maintaining in the medium without serum. Medium containing 20% FBS was added to the lower chamber as a chemoattractant. Subsequently, the cells were incubated at 37°C for 24 h. Noninvading cells were removed while the cells migrated to the bottom of the membrane were fixed with cold methanol and stained with 0.1% crystal violet for 20 min. The stained cells were captured under a microscope in five random fields with 100x magnification, and the average number of migratory cells was taken. All the experiments were repeated 3 times.

RETRACTED

### 2.6. Luciferase Reporter Assay

We performed luciferase reporter assay to investigate whether there is a direct transcript relationship between miR-509-5p and TRIB2 as well as TRIB2 and p21. Firstly, the 3′-TUR of TRIB2 was amplified and cloned to the restrictive site between Xho I and Bgl II of pGL6-miR. Subsequently, the site mutation kit (Beyotime Biotechnology, Shanghai, China) was used to mutate the 3′-TUR site of TRIB2 targeted with miR-509-5p. A similar procedure was conducted to produce a p21 mutant version. After that, 5 × 10^3^ cells were seeded into the 96-well plates and then transfected with the wild-type or mutated report vector or the negative control for 48 h. The firefly luciferase activity was measured according to the dual luciferase reporter assay manually (Beyotime Biotechnology, Shanghai, China). All the experiments were repeated 3 times.

### 2.7. Western Blot

The total protein of the cultured cells was extracted using the radioimmunoprecipitation assay buffer (Beyotime Biotechnology, Shanghai, China) mixed with protease inhibitor cocktail (Thermo Fisher Scientific, Inc.). After the total protein concentrations of the cell lysates were measured using the Bicinchoninic Acid Protein Assay kit (Thermo Fisher Scientific, Inc.), 20 *μ*g protein of each sample was electrophoresed on the SDS-PAGE gel and then transferred onto polyvinylidene fluoride (PVDF) membranes (Millipore Sigma, USA). The membranes were then blocked with 5% nonfat milk in TBST at room temperature for 1 h and then incubated at 4°C overnight with primary antibody against TRIB2 (Abcam, ab117981, 1 : 1000), p21 (Abcam, ab129520, 1 : 1000), and GADPH (Abcam, ab181602, 1 : 1000). Washing twice with TBST, the membranes were incubated with second antibody at room temperature for 1 h. Antibody binding was detected via enhanced chemiluminescence and the band density was analyzed with software. All the experiments were repeated 3 times.

### 2.8. Statistical Analysis

The results were presented as mean ± standard deviation after the analysis with SPSS, version 19.0. One-way ANOVA or independent *t*-test was used to calculate the *P* value. *P* < 0.05 was considered a statistically significant difference.

## 3. Results

### 3.1. The Expression of miR-509-5p Was Decreased in the OS Tissues and Cell Lines

The expression date of miR-509-5p in OS tissues was evaluated from GEO database (https://www.ncbi.nlm.nih.gov/geo/query/acc.cgi?acc=GSE28423). The GEO2R tools from the website were used to compare the expression of miR-509-5p in normal tissues and OS tumor tissues. As we can see in Figure 1(a), the expression of miR-509-5p in the OS tissues was decreased significantly compared with the normal tissues. To validate the result with the tissues got from our hospital, we performed RT-PCR experiments to investigate the expressions of miR-509-5p in 14 paired OS tissues and adjacent normal tissues. As a result, the expression of miR-509-5p was decreased in 11 out of the 15 OS tissues compared with the paraneoplastic tissues (Figure 1(b)). In addition, the miR-509-5p expression was further investigated in various OS cell lines, including U2OS, HOS, Saos-2, and MG-63. As shown in Figure 1(c), the miR-509-5p was downregulated in these OS cell lines compared with normal human osteoblast cell line (NHOst). In conclusion, these results suggested that miR-509-5p was ectopically decreased in the OS tissues and cells.

RETRACTED

### 3.2. miR-509-5p Could Inhibit Proliferation and Invasion of the OS Cells

To investigate the biological function of miR-509-5p in OS, the cell lines U2OS and HOS were transfected with miR-509-5p overexpressing vector HIVH1-miR-509-5p and corresponding NC. The transfection efficiency was detected by RT-PCR; as shown in Figure 2(a), the expression level of miR-509-5p after overexpression was increased remarkably. The result of CCK-8 assay suggested that the proliferation potential of U2OS and MG-63 transfected with HIVH1-miR-509-5p was markedly decreased compared with the NC-miR (Figure 2(b)). Transwell assay result showed that the invasion ability of the miR-509-5p overexpression group decreased significantly compared with the NC group, suggesting that miR-509-5p could inhibit the invasion ability of OS cells (Figure 2(c)). In conclusion, these data revealed that miR-509-5p could act as a tumor suppressor and inhibit the proliferation and invasion of OS cells.

### 3.3. TRIB2 Is Upregulated in OS Tissues and Is a Direct Target of miR-509-5p

We continue to investigate GEO databases and finally found 2 databases (GSE39055 and GSE11416) presenting the expression of mRNA in OS tissues and normal tissues nearby. We compared the mRNA expression of each database to find out the upregulated gene in OS and finally get a cohort of 320 genes in GSE39055 and 53 genes in GSE11416. And as shown in Figure 3(a), we find that TRIB2 is upregulated in OS tissues from both GSE databases. This indicated that TRIB2 may be upregulated in most OS tissues and may function as an oncogene in OS.

It is well recognized that miRNA participated in various physiological activities through binding to the mRNA 3′-UTR of the target gene. In order to identify the targeted mRNA of miR-509-5p, the TargetScan (http://www.targetscan.org) database was used to predict the potential target. As a result, TRIB2 was predicted to be a potential target of miR-509-5p (Figure 3(b)). RT-PCR was conducted to detect the mRNA level of TRIB2 in OS tissues for further validation. The result showed that, compared with the normal control group, the expression of TRIB2 was greatly overexpressed in OS tissues, which was negatively correlated with the miR-509-5p level (Figure 3(c)). As expected, the TRIB2 mRNA increased significantly in the OS cell lines U2OS, HOS, Saos-2, and MG-63 compared with the NHOst (Figure 3(d)). The subsequent western blot further confirmed that the protein expression of TRIB2 decreased in the same cell lines (Figure 3(e)). To further confirm whether miR-509-5p may target TRIB2 in OS, we upregulated the miR-509-5p expression by the vector described above and found a markedly reduced expression of TRIB2 in both mRNA and protein level in U2OS and HOS cells (Figure 3(f)). Taken together, these results imply that miR-509-5p targets TRIB2 in OS cells.

RETRACTED

### 3.4. Knockdown of TRIB2 Could Inhibit the Malignant Capacity of OS Cells

In order to confirm whether TRIB2 is responsible for the tumor suppressive role of miR-509-5p in OS cells, we knock down the TRIB2 through small interfering RNA in the U2OS and HOS cells. The silence effect was assessed by western blot (Figure 4(b)). As a result, the proliferation and invasion ability of both cell lines decreased markedly after TRIB2 was silenced (Figures 4(c) and 4(d)), which was very close to the effect of miR-509-5p overexpressing.

### 3.5. p21 May Be the Downstream Effect of miR-509-5p Targeting TRIB2

The luciferase reporter assay was performed to validate whether there is a direct interaction between miR-509-5p and TRIB2. The suppositional binding site of the 3′-UTR in TRIB2 was cloned into the luciferase reporter vector as a wild-type version (pMir-Wt) while a deletion of 8 bp in the seed region of the 3′-UTR was constructed as a mutant version (pMir-Mut). The results show that attenuated luciferase activities were observed in the U2OS and HOS cells cotransfected with pMir-Wt and miR-509-5p overexpression vector (Figure 4(a)), which indicated miR509-9p binding to the 3′-UTR of TRIB2 directly.

As the downstream effect of miR-509-5p targeting TRIB2 remains unknown, we conducted western blot in the U2OS and HOS cells and the results showed that the expression of p21 protein increased significantly after the TRIB2 was knocked down by small interfering RNA (Figure 4(e)). In addition, as shown in Figure 4(f), a markedly enhanced luciferase activity was observed in the cells cotransfected with si-TRIB2 and p21 mutant version (p21-luc). In conclusion, these results implied that p21 may be the downstream effect of miR-509-5p targeting TRIB2.

RETRACTED

## 4. Discussion

As the most common malignant primary bone tumor, OS remains a serious threat to the children despite the progress in treatment strategy. Therefore, it is urgent and vital to find a new therapeutic strategy to suppress OS. In the past decades, miRNA has been well demonstrated to participate in tumor progression through regulating the expression of oncogenes and tumor suppressors [13]. miR-509-5p is a member of miR-509 family [14], which has been reported to act as a tumor suppressive role in renal cell carcinoma (RCC) [15] and cervical cancer [16]. However, the function and mechanism of miR-509-5p in OS have never been investigated.

In the present study, we observed a markedly downregulation of miR-509-5p in the OS tissues compared with the adjacent normal tissues. Similar results in the OS cell lines were found to further confirm the hypothesis that miR-509-9p may be a tumor suppressor gene. Subsequently, we conducted the in vitro cell culture to investigate the biological function of miR-509-5p in the progression of OS. The results revealed that overexpression of miR-509-5p inhibited OS cell proliferation and invasion, which indicated that miR-509-5p is an OS suppressor gene. We further investigated the underlying mechanism of how the miR-509-5p inhibits the OS progression. Although miR-509-5p should have many targets, for example, MDM2, SOD2, FOXP1, etc., we identified TRIB2 as a direct target of miR-509-5p while it is a putative oncogene that is also highly expressed in OS tissues. Furthermore, the result of subsequent luciferase reporter gene suggested that TRIB2 inhibited the bioactivity of a well-recognized tumor suppressor gene, p21, through blocking its transcriptional activity [17]. In conclusion, miR-509-5p acts as an antitumor gene in OS through inhibiting the expression of TRIB2, an oncogene that decreased the expression of p21 and attenuated the antitumor function, thus increasing cancer risk and accelerating the OS progression.

As a member of the tribble family, tribbles homolog 2 (TRIB2) is a mitosis blocker that regulates embryo and germ cell development [18]. It has been reported that, as a scaffold protein [19], TRIB2 plays a critical role in various biological processes as well as in pathological conditions, especially in tumor development [20, 21]. For instance, the overexpression of TRIB2 may accelerate the acute myeloid leukemia (AML) through activating C/EBP*α* pathway [22]; in liver cancer, TRIB2 promoted cell proliferation and transformation via improving the stabilization of YAP through the E3 ubiquitin ligase *β*TrCP [23]. To extensively study the mechanisms related to the downstream effect of TRIB2-mediated regulation, we found a directed connection between TRIB2 and p21. Although it is well known that p21 is mainly regulated by p53 at the transcription level [24], there are multiple transcription factors such as BRCA1, Smad3, AP4, and c-myc that also control the expression of p21 [25–27]. Here, we reported that TRIB2 negatively regulates the promoter of p21 and thus inhibits the antitumor effect of p21, resulting in the progression of OS. However, further studies are still needed to explore the exact mechanism of how TRIB2 impacts the bioactivity of p21 (Figure 5).

RETRACTED

In conclusion, our study demonstrated that the expression of miR-509-5p was significantly decreased in OS tissue and cell lines. Simultaneously, we also identified that TRIB2 was a direct and functional target of miR-509-5p, which thus negatively regulates the antitumor effect of p21. Taken together, our study indicated that restoration of miR-509-5p or knockout of TRIB2 may be the potential preventive and/or therapeutic interventions for OS.

## Figures and Tables

**Figure 1:** miR-509-5p expression in OS tissues and cell lines. (a) The GEO2R result from the GEO database GSE28423 indicated that the expression of miR-509-5p in the local OS tissues and the metastasized tissues decreased significantly compared with the normal tissues. (b) miR-509-5p relative expressions in 15 pairs of OS tissues and adjacent normal tissues were detected via q-PCR. *N* = 5. *P* < 0.0001 vs. normal tissues. (c) miR-509-5p expressions in OS cell lines (U2OS, HOS, Saos-2, and MG-63) were detected via q-PCR. *N* = 5. ^*∗*^*P* < 0.01, ^*∗∗*^*P* < 0.0001 vs. NHOst cells.

**Figure 2:** miR-509-5p inhibits OS cell lines proliferation and invasion. (a) The relative expression of miR-509-5p in U2OS and MG-63 cell lines following transfection with miR-509-5p overexpressing vector or control. (b) The cell proliferation ability of U2OS and MG-63 transfected with miR-509-5p overexpressing vector or control was detected by CCK-8 assay. (c) The invasion ability of U2OS and MG-63 cells transfected with miR-509-5p overexpressing vector or control was detected by Transwell assay. ^*∗*^*P* < 0.01, ^*∗∗*^*P* < 0.0001 vs. control.

**Figure 3:** miR-509-5p targets TRIB2 in OS cells. (a) TRIB2 was found to be the unique upregulated gene in both GSE39055 and GSE11416 gene expression profiles. (b) The putative binding sites of miR-509-5p in 3′-UTR of TRIB2. (c) The relative expressions of TRIB2 in OS tissues were detected by q-PCR. TRIB2 level was negatively correlated with the miR-509-5p level in OS tissues. ^*∗∗*^*P* < 0.0001 vs. control. (d, e) The mRNA and protein expressions of TRIB2 in OS cell lines (NHOst, U2OS, HOS, Saos-2, and MG-63) were detected via q-PCR and western blot, respectively. ^*∗*^*P* < 0.01, ^*∗∗*^*P* < 0.0001 vs. NHOst. (f) The mRNA and protein expression of TRIB2 in U2OS and HOS cell lines following transfection with miR-509-5p overexpressing vector or control. ^*∗∗*^*P* < 0.0001 vs. control.

RETRACTED

**Figure 4:** p21 may be the downstream effect of miR-509-5p targeting TRIB2. (a) Luciferase reporter gene assay was conducted to assess whether miR-509-5p directly targeted TRIB2 in cells cotransfected with pMir-Wt or pMir-Mut and either miR-509-5p overexpression vector or NC-miR. The mean of the results from cells transfected with expression control vector and pMir-con was set as 100. ^*∗∗*^*P* < 0.0001 vs. pMir-Wt. (b) The silence effect was detected by western blot after U2OS and HOS cell lines were transfected with si-TRIB2. (c, d) Cell proliferation and invasion ability of U2OS and HOS cells transfected with si-TRIB2 or si-NC were detected by CCK-8 or Transwell assay, respectively. (e) The p21 expressions of U2OS and HOS cells transfected with si-TRIB2 or si-NC were detected by western blot. (f) Luciferase reporter gene assay showed that a markedly enhanced luciferase activity was observed in the cells cotransfected with si-TRIB2 and p21 mutant version (p21-luc).

**Figure 5:** The miR-509-5p hypothesis. miR-509-5p binding to the 3′-UTR region of TRIB2 sequentially inhibits the bioactivity of the tumor suppressor gene p21, suggesting that miR-509-9p is an OS suppressor.

## Data Availability

The data used to support the findings of this study are available from the corresponding author upon request.

## References

[1] Valery P. C., Laversanne M., Bray F. (2015). Bone cancer incidence by morphological subtype: a global assessment. *Cancer Causes & Control*.

[2] Toki S., Kobayashi E., Yoshida A. (2019). A clinical comparison between dedifferentiated low-grade osteosarcoma and conventional osteosarcoma. *The Bone & Joint Journal*.

[3] Wachtel M., Schäfer B. W. (2010). Targets for cancer therapy in childhood sarcomas. *Cancer Treatment Reviews*.

[4] Zhang C., Hu J., Zhu K., Cai T., Ma X. (2018). Survival, complications and functional outcomes of cemented megaprostheses for high-grade osteosarcoma around the knee. *International Orthopaedics*.

[5] Dong X. Q., Zhang Y. H., Shang X. Q., Zeng Y. J. (2019). Effects of miR-101 on the proliferation and apoptosis of gastric mucosal epithelial cells via Nrf2/ARE signaling pathway. *European Review for Medical and Pharmacological Sciences*.

[6] Shao Y., Liu X., Meng J., Zhang X., Ma Z., Yang G. (2019). MicroRNA-1251-5p promotes carcinogenesis and autophagy via targeting the tumor suppressor TBCC in ovarian cancer cells. *Molecular Therapy*.

RETRACTED

[7] Yang Y. J., Luo S., Wang L. S. (2019). Effects of microRNA-378 on epithelial-mesenchymal transition, migration, invasion and prognosis in gastric carcinoma by targeting BMP2. *European Review for Medical and Pharmacological Sciences*.

[8] Yu Y., Zhao J. D., Yang H. (2019). MiR-299-3p inhibits proliferation and invasion of cervical cancer cell via targeting TCF4. *European Review for Medical and Pharmacological Sciences*.

[9] Zhang Z. F., Wang Y. J., Fan S. H. (2017). MicroRNA-182 downregulates Wnt/beta-catenin signaling, inhibits proliferation, and promotes apoptosis in human osteosarcoma cells by targeting HOXA9. *Oncotarget*.

[10] Duan J., Liu J., Liu Y., Huang B., Rao L. (2017). miR-491-3p suppresses the growth and invasion of osteosarcoma cells by targeting TSPAN1. *Molecular Medicine Reports*.

[11] Xu Q., Cheng L., Chen J., Lu W., Wang P. (2019). miR-376a inhibits the proliferation and invasion of osteosarcoma by targeting FBXO11. *Human Cell*.

[12] Zhou Y., Huang Z., Wu S., Zang X., Liu M., Shi J. (2014). miR-33a is up-regulated in chemoresistant osteosarcoma and promotes osteosarcoma cell resistance to cisplatin by down-regulating TWIST. *Journal of Experimental & Clinical Cancer Research*.

[13] Zhu K.-P., Zhang C.-L., Ma X.-L., Hu J.-P., Cai T., Zhang L. (2019). Analyzing the interactions of mRNAs and ncRNAs to predict competing endogenous RNA networks in osteosarcoma chemo-resistance. *Molecular Therapy*.

[14] Song Y. H., Wang J., Nie G. (2017). MicroRNA-509-5p functions as an anti-oncogene in breast cancer via targeting SOD2. *European Review for Medical and Pharmacological Sciences*.

[15] Zhang W.-B., Pan Z.-Q., Yang Q.-S., Zheng X.-M. (2013). Tumor suppressive miR-509-5p contributes to cell migration, proliferation and antiapoptosis in renal cell carcinoma. *Irish Journal of Medical Science*.

[16] Ren Z.-J., Nong X.-Y., Lv Y.-R. (2014). Mir-509-5p joins the Mdm2/p53 feedback loop and regulates cancer cell growth. *Cell Death & Disease*.

[17] Hou Z., Guo K., Sun X. (2018). TRIB2 functions as novel oncogene in colorectal cancer by blocking cellular senescence through AP4/p21 signaling. *Molecular Cancer*.

[18] Grosshans J., Wieschaus E. (2000). A genetic link between morphogenesis and cell division during formation of the ventral furrow in Drosophila. *Cell*.

[19] Sakai S., Miyajima C., Uchida C., Itoh Y., Hayashi H., Inoue Y. (2016). Tribbles-related protein family members as regulators or substrates of the ubiquitin-proteasome system in cancer development. *Current Cancer Drug Targets*.

RETRACTED

[20] Do E. K., Park J. K., Cheon H. C. (2017). Trib2 regulates the pluripotency of embryonic stem cells and enhances reprogramming efficiency. *Experimental & Molecular Medicine*.

[21] Hua F., Mu R., Liu J. (2011). TRB3 interacts with SMAD3 promoting tumor cell migration and invasion. *Journal of Cell Science*.

[22] Keeshan K., He Y., Wouters B. J. (2006). Tribbles homolog 2 inactivates C/EBP*α* and causes acute myelogenous leukemia. *Cancer Cell*.

[23] Wang J., Park J.-S., Wei Y. (2013). TRIB2 acts downstream of wnt/TCF in liver cancer cells to regulate YAP and C/EBP*α* function. *Molecular Cell*.

[24] Kato S., Han S.-Y., Liu W. (2003). Understanding the function-structure and function-mutation relationships of p53 tumor suppressor protein by high-resolution missense mutation analysis. *Proceedings of the National Academy of Sciences*.

[25] Elbendary A., Berchuck A., Davis P. (1994). Transforming growth factor beta 1 can induce CIP1/WAF1 expression independent of the p53 pathway in ovarian cancer cells. *Cell Growth & Differentiation*.

[26] Somasundaram K., El-Deiry W. S. (1997). Inhibition of p53-mediated transactivation and cell cycle arrest by E1A through its p300/CBP-interacting regionSelfcloseTable. *Oncogene*.

[27] Wu S., Cetinkaya C., Munoz-Alonso M. J. (2003). Myc represses differentiation-induced p21CIP1 expression via Miz-1-dependent interaction with the p21 core promoter. *Oncogene*.

